# Cynarin suppresses gouty arthritis induced by monosodium urate crystals

This article has been retracted.

**DOI:** 10.1080/21655979.2022.2072055

**Published:** 2022-05-12

**Authors:** Changgui Wu, Shaohua Chen, Yang Liu, Bo Kong, Wei Yan, Tao Jiang, Hao Tian, Zhaoyi Liu, Qi Shi, Yongjun Wang, Qianqian Liang, Xiaobing Xi, Hao Xu

**Affiliations:** a Department of Orthopaedics, Shanghai Ruijin Hospital, Shanghai Jiao Tong University School of Medicine, Shanghai, China; b Longhua Hospital, Shanghai University of Traditional Chinese Medicine, Shanghai, China; c Tianshan Hospital of Traditional Chinese Medicine, Shanghai, China; d Shanghai Guanghua Hospital of Integrated Traditional Chinese and Western Medicine, Shanghai, China; e Key Laboratory of Theory and Therapy of Muscles and Bones, Ministry of Education (Shanghai University of Traditional Chinese Medicine), Shanghai, China

**Keywords:** Cynarin, gouty arthritis, JNK, NF-κB, NLRP3 inflammasomes

## Abstract

The study is aimed to determine the effects of cynarin (Cyn) on mice with gouty arthritis (GA) induced by monosodium urate (MSU). We measured swelling in the hind paws of mice *in vivo* using Vernier calipers and ultrasound. The liver, kidney, and hind paws were stained with hematoxylin-eosin, and M1 type macrophages were detected in the hind paws using anti-F4/80 and anti-iNOS antibodies. The mRNA expression of inflammatory factors in bone marrow-derived macrophages (BMDMs) and in the hind paws was detected via quantitative reverse transcription-polymerase chain reaction (qRT-PCR). Nucleotide-binding oligomerization domain (NOD)-like receptor (NLR) family pyrin domain containing 3 (NLRP3) inflammasomes and the nuclear factor kappa B (NF-κB) and mitogen-activated protein kinase (MAPK) pathways were analyzed via western blotting. Cyn was detected *in vitro* using Cell Counting Kit-8 (CCK-8). Cyn treatment reduced hind paw swelling and M1 macrophage infiltration, suppressed the mRNA expression of inflammatory factors, and inhibited NLRP3 inflammasome activation *in vivo*, in addition to inhibiting the phosphorylation of IKKa/β, p65, and c-Jun NH 2-terminal kinase (JNK). Furthermore, Cyn exerted anti-inflammatory and anti-swelling effects in mice with GA by regulating the NF-κB and JNK pathways and NLRP3 inflammasomes.

## Highlights

- Cynarin relieved the symptoms of gouty arthritis induced by MSU *in vivo*.
- Cynarin inhibited MSU-induced inflammatory response in gouty arthritis by reducing the infiltration of M1 type macrophages.
- Cynarin exerted an effect on gouty arthritis by regulating NF-κB, JNK pathways and NLRP3 inflammasome.

## Introduction

Gout is a metabolic disease and a common cause of inflammatory arthritis [1,2]. Epidemiological studies show that the prevalence of gout is 0.6% in developed and 1.1% in China [3,4]. The prevalence is 1.5% among men and 0.9% for women [4]. Disorders of the purine catabolic pathway cause hyperuricemia wherein serum urate levels consistently exceed in limit of 7.0 mg/dL [2]. Long-term untreated hyperuricemia can lead to the formation and deposition of monosodium urate (MSU) crystals in joints and soft tissues, thereby causing damage and inflammation, and eventually induce gouty arthritis (GA) [5–10]. The onset of GA is characterized by severe pain, swelling, fever, and redness and advanced gout can be clinically detected tophi by ultrasound [11–13].

Macrophage activation is closely related to the onset of GA [14,15]. Macrophages are important immune cells and have remarkable phagocytosis and adhesion functions; they play vital roles in the host defense system by infiltrating the sites of inflammatory responses and phagocytosing of foreign bodies [16]. inflammatory MSU causes chemotactic macrophages to accumulate in the joints and surrounding tissues where they phagocytose MSU [2,17]. Thereafter, intracellular inflammatory factor secretion activates the NLRP3 inflammasome and NF-κB signaling pathways [1,2,18]. MSU crystals injected into the hind paws of mice cause GA, inflammatory cell infiltration and the release of inflammatory factors [19,20].

Clinically diagnosed GA is usually treated with uric acid excretion drugs, xanthine oxidase inhibitors (allopurinol and benzbromarone), anti-inflammatory drugs (colchicine, indomethacin, and indomethacin), hormones and other agents [21,22]. However, these agents are associated with side effects such as gastrointestinal, liver, and kidney toxicity; hence, their long-term application is restricted [23]. Interest in natural herbs has increased owing to advantages such as wide sources, good effects, low price, and low toxicity [24,25]. Compound Fu Rong Ye Babu Ointment used to our department is clinically effective against GA, and cynarin (Cyn) was identified by screening compound prescriptions that were analyzed using Traditional Chinese Medicine Systems Pharmacology (TCMSP) database, literature search and qRT-PCR. However, the effect of Cyn on MSU-induced GA in mice remain unclear.

We speculated that Cyn would exert anti-inflammatory and anti-swelling effects against GA in mice. Therefore, we aimed to determine whether Cyn inhibits the symptoms in mice with GA induced by MSU.

## Materials and methods

### Animals

C57BL/6 male mice were used for GA experiments [19,26]. The study used 30 C57BL/6 j male mice (22 ± 3 g) aged 6–8 weeks, provided by Shanghai Jie Sijie Experimental Animal Co., Ltd. (license number #SCXK2018-0004). The mice lived in an environment with suitable temperature, humidity, and sufficient water and food. All animal experiments were performed under the approval of the Animal Ethics Committee of Shanghai University of Traditional Chinese Medicine (Shanghai, China). The ethics number is PZSHUTCM201211002.

### Main instruments and reagents

Main instruments: Vernier caliper (Meinaite, Germany), Ultrasound imaging equipment (Vevo 3100), dehydrator, embedding machine, slicer, spreader (Leica, Germany), automatic tissue scanner (VS120, Olympus).

Main reagents: Cynarin (Chengdu Pufei De Biotechnology, 17041106), xylene (Sinopharm, 10023418), Ethylenediamine tetraacetic acid (Sinopharm. 10009617), 75%Ethanol (Sinopharm, 80176961), Absolute ethanol (Sinopharm, 10009218), Hematoxylin(sigma, H3136), Eosin Y (sigma, E4009), Monosodium Urate (sigma, U2875), Bovine Serum Albumin (Aladdin, B265994),Anti-F4/80 antibody (Abcam, ab6640), Macrophage-stimulating factor (MCSF) (Peprotech, 315–02), Anti-iNOS antibody (Abcam, ab3523), VECTASHIELD Mounting Medium with DAPI (Vectorlabs, H-1200), Trypsin antigen repair solution (Leagene Biotechnology, IH0310), Cell Counting Kit-8 (Dojindo laboratories, CK04), PrimeScript™ RT Reagent Kit (TaKaRa, RR037A), qPCR SYBR Green Master Mix (YESEN, 11201ES03), p-p65 antibody (CST, 3033), p65 antibody (CST, 8242), GAPDH antibody (sigma, G9545), p-p38 antibody (CST, 4511), p-IKKa/β antibody (CST, 2697),Anti-rabbit antibody (CST, 7074), p-JNK antibody (CST, 4668), p-ERK1/2 antibody (CST, 4370), Caspase 1/p20/p10 antibody (Proteintech, 22915-1-AP), Anti-NLRP3 antibody (Abcam, ab263899), Anti-IL-1β antibody (Abcam, ab200478).

### Drug administration

A 3% suspension of MSU in distilled water (0.6 mg/20 μL) was injected into the hind paws of C57BL/6 male mice to construct GA models [19,20]. The mice were randomly assigned to groups (n = 10 each) that received phosphate-buffered saline (PBS; 20 μL injected into a hind paw, followed by intraperitoneal [i.p.] injection of 200 μL normal saline), MSU (20 μL of 3% MSU injected into the hind paw, followed by i.p. injection of 200 μL normal saline), or MSU+Cyn (3% MSU injected into the hind paw, followed by i.p. injection of 200 μL Cyn [25 mg/kg] i.p.) for 7 days (Figure 1) [19,27].

**Figure 1.** The time chart of induction and treatment process in mice with gouty arthritis

### Measurement of hind paw thickness in mice

The thickness of hind paws was measured daily for seven days using a Vernier caliper placed perpendicular to the paws [19].

### Ultrasound imaging

Ultrasound can detect tophi in patients with advanced gout [13]. Therefore, we analyzed the hind paws of all mice using ultrasound imaging in B mode after seven days of treatment. The mice were placed on the ultrasound workbench and adjusted to the optimal position in which their hind paws were completely exposed and remained parallel to the ultrasound probe.

### Tissue preparation

The mice were euthanized immediately after ultrasound images were acquired. The liver, kidney, and hind paws were excised and placed in a 4% tissue fixative for 24 h; then, the liver and kidneys were dehydrated and embedded in paraffin. The hind paws were decalcified in 13% disodium ethylenediaminetetraacetic acid that was replaced every three days for 30 days; then, the paws were dehydrated and embedded.

### Hematoxylin-eosin (HE) staining

As previously stated, HE staining was performed on mouse tissues [19]. The paraffin-embedded livers, kidneys, and hind paws were heated at 60°C for 1 h, deparaffinized thrice with xylene, and hydrated in a series of decreasing concentrations of ethanol. The tissue sections were stained with hematoxylin for 1 min, placed in 1% hydrochloric acid in ethanol for 1 min, washed, and then immersed in 2% ammonia water for 5 s, followed by eosin for 1 min. The sections were dehydrated in a series of increasing concentrations of ethanol and rendered transparent with xylene. Tissue sections were mounted with neutral resin and heated at 60°C for 2 h.

### Immunofluorescence staining

Anti-F4/80 (diluted 1:300) and anti-iNOS (diluted 1:400) were the primary antibodies, and the secondary antibody was (diluted 1:500). Hind paw tissue slides, after being heated at 60°C for 1 h, were deparaffinized in xylene and then hydrated with a decreasing gradient of ethanol concentrations. Antigens were retrieved using trypsin for 7 min, then, nonspecific antigen binding was blocked with 5% bovine serum albumin (BSA) for 1 h. The sections were incubated with anti-F4/80 and anti-iNOS antibodies overnight at 4°C, followed by secondary antibody for 1 h in the dark, and then mounted with an anti-fluorescence quencher (VECTASHIELD Mounting Medium with DAPI (Vectorlabs)) [28].

### Cells culture

Bone marrow-derived macrophages (BMDMs) were extracted from the femurs and tibias of euthanized 6–8-week-old male C57BL/6 mice into RPMI 1640 complete medium (containing 10% fetal bovine serum and 1% double antibodies (penicillin and streptomycin)), passed through 40 μm filters, and lysed with red blood cell lysate. The lysates were centrifuged, resuspended, and inoculated into 6 cm Petri dishes containing MCSF solution (containing 1640 complete medium and 20 ng/ml MCSF) [28]. Half of the culture medium was replaced 2, 4, and 6 days later, and the cells were cultured for 7 days [28].

### CCK-8 assays

Cell viability was evaluated as described by the manufacturer of CCK-8 (Dojindo laboratories). The cultured BMDMs were seeded into 96-well plates and left overnight. On the following day, the medium was replaced with RPMI 1640 complete medium with or without Cyn, and the cells were incubated for 24 h. The medium was again replaced with RPMI 1640 complete medium containing 10% CCK-8, and the cells were cultured for 2–4 h. Cell viability was examined using a microplate reader.

### Quantitative RT-PCR

The cultured BMDMs were incubated with lipopolysaccharide (LPS, 500 ng/mL), MSU(300 μg/mL), or Cyn (290 μM) [22,29]. Total RNA extracted from the processed BMDMs and fresh hind paws of mice, using Trizol, was thoroughly mixed with chloroform, centrifuged, and the supernatant was collected. The pellets were resuspended in isopropanol and centrifuged. The supernatant was discarded, following which the pellet was resuspended in 70% absolute ethanol and centrifuged; the ethanol supernatant was discarded. The resultant RNA was reverse transcribed into cDNA, which was amplified via qRT-PCR under the following conditions: 95°C for 5 min, followed by 40 cycles at 95°C for 10 sec and 60°C for 30 sec. Data from three independent experiments were used to determine mRNA expression using the 2^^(−ΔΔCT)^ method. Table 1 shows the PCR primers.

**Table 1.** Sequences of primers used in the qRT-PCR

Primers	Sequences (5’ to 3’)
IL-1β Forward	CTGGTACATCAGCACCTCAC
IL-1β Reverse	AGAAACAGTCCCAGCCCATAC
IL-6 Forward	TGTATGAACAACGATGATGCACTT
IL-6 Reverse	ACTCTGGCTTTGTCTTTCTTGTTATCT
TNF-α Forward	AGTGACAAGCCTGTAGCCC
TNF-α Reverse	GAGGTTGACTTTCTCCTGGTAT
iNOS Forward	AACGGAGAACGTTGGATTTG
iNOS Reverse	CAGCACAAGGGGTTTTCTTC
β-actin Forward	CGTTGACATCCGTAAAGACC
β-actin Reverse	TAGGAGCCAGAGCAGTAATC

### Western blotting

As described in the previous study, the mechanism of drugs on GA can be elucidated by WB experiments [27]. p-p65, p65, p-p38, p-IKKa/β, p-JNK, p-ERK1/2, Caspase 1/p20/p10, Anti-NLRP3 antibody and secondary antibody were all diluted 1:1000. Anti-IL-1β antibody was used at a concentration of 2ug/ml and GAPDH antibody was diluted 1:5000. The BMDMs and mouse hind paws were lysed with RIPA lysis buffer (Beyotime Biotechnology, P0013C). Protein concentrations were measured using BCA Protein Assay Kits (Beyotime Biotechnology, P0010). Next, 1.8 and 9.8 μg/μL of proteins were resolved via electrophoresis device (BIO-RAD) and blotted onto membranes. Nonspecific protein binding on the membranes was blocked using the quickBlock™ Blocking Buffer (Beyotime Biotechnology, P0252); then, the membranes were incubated with primary antibodies at 4°C overnight, followed by secondary antibodies, in the dark. Color was then developed using a developer solution. Integrated density was determined from three independent experiments using ImageJ 5.0

### Statistical analysis

GraphPad Prism 8.0.1, ImageJ, and SPSS 20.0 software were used for statistical analysis. When the normality test was met and the variances were uniform, the analysis of variance was used for comparison between multiple groups, and the pairwise comparisons were based on the Tukey analysis after the analysis of variance. When the data was repeatedly measured, repeated measures analysis of variance was used. The data were all expressed as mean ± standard deviation (SD). The validity test adopted two-sided test, and the test level was α = 0.05, and the difference was statistically significant with *p* < 0.05.

## Results

We speculated that Cyn would exert anti-inflammatory and anti-swelling effects against GA in mice. We therefore explored the effects and mechanisms of Cyn against GA in mice and in BMDMs stimulated with MSU. We found that Cyn effectively alleviated GA in mice by regulating the NF-κB and JNK pathways and NLRP3 inflammasomes.

### Cynarin treatment reduced hind paw swelling in mice with GA

Thirty C57BL/6 mice were randomly divided into three groups that received PBS (control), MSU, or MSU+Cyn for seven days (Figure 1). The hind paws were significantly less swollen in the MSU+Cyn group than in the MSU group (Figure 2(a,b)) and more swollen in the MSU and MSU+Cyn groups than in the PBS group.

**Figure 2.** Cynarin reduced hind paws swelling in mice with gouty arthritis. (a) After 7 days, changes in hind paws of mice with gouty arthritis. (b) The hind paws of mice were measured and recorded daily using vernier calipers. (c) After 7 days, the swelling of the hind paws of mice was measured using an ultrasound, and the results were displayed in B-mode and 3D-mode. (d) Data were collected using ultrasound software. Data were shown as mean ± standard deviation (SD) of ten mice per group. *p<0.05, **p<0.01, ***p<0.001 VS. MSU group. ^###^*p*<0.001 VS. PBS group.

One week later, ultrasound revealed more swelling in hind paws from the MSU and MSU+Cyn groups than in those from the PBS group. The hind paws were significantly smaller in the MSU+Cyn group than in the MSU group (Figures 2(c,d)).

### Cyn did no adverse effects on the liver and kidney of mice

We stained the kidney and liver tissues of mice with HE to determine whether Cyn exerts any deleterious effects. The kidney and liver tissues of all groups of mice were structurally complete, boundaries were obvious and cells in both the organs were not degenerated or necrotic, and glomeruli were clearly visible in the cortices of the kidneys (Figure 3(a,b)).

**Figure 3.** The effect of Cyn on kidney and liver tissues. (a, b) Hematoxylin-eosin staining of kidney and liver tissues. The scale in the figure is 50μm.

### Cynarin treatment reduced M1 macrophage infiltration in mice with GA

The hind paws of each group of mice were stained with HE. Inflammatory cell infiltration was not evident in the soles of hind paws and synovia of metatarsophalangeal joints in the PBS group. In contrast, the MSU and MSU+Cyn groups both had inflammatory cell infiltration, but the extent was greater in the MSU group (Figure 4(a,b)). The proportions of inflamed areas were significantly higher in the MSU group than in the PBS group and significantly lower in the MSU+Cyn group than in the MSU group (Figure 4(c)).
**Figure:**

**Figure 4.** Cynarin inhibited the infiltration of inflammatory cells. (a) The hind paws of mice were stained with hematoxylin and eosin (HE). the scale in the figure is 500μm and 200μm. (b) Synovial tissues of mouse hind paw metatarsophalangeal joint. the scale in the figure is 50μm. (c) Statistics and analysis of the proportion of inflammatory area on the hind paws after HE staining. (d) The hind paws of the mice were stained with immunofluorescence. the scale in the figure is 20μm. (e) Statistics and analysis of the percentage of positive area on the hind paws of mice after immunofluorescence staining. Data were shown as mean ± standard deviation (SD) of ten mice per group. ***p<0.001 VS. MSU group, ^###^*p*<0.001 VS. PBS group.

Immunofluorescence staining revealed no inflammatory macrophage infiltration in the hind paws of mice in the PBS group. In contrast, inflammatory macrophage infiltration was observed in both the MSU and MSU+Cyn groups but was significantly more evident in the MSU group (Figure 4(d)). The proportions of positively stained areas were higher in the MSU and MSU+Cyn groups than in the PBS group, but to a lesser extent in the MSU+Cyn group (Figure 4(e)).

### Cynarin inhibited the relative mRNA expression of inflammatory factors in M1 macrophages

We incubated BMDMs with Cyn for 24 h and then evaluated cell viability using the CCK8 kit. Cynarin ≤ 387 μM was not toxic to BMDMs (Figure 5(a)). Monosodium urate crystals activate mononuclear macrophages to secrete numerous inflammatory factors [1,28,30]. Inhibition of inflammatory factor secretion is a promising strategy for treating GA [2]. Therefore, we assessed the therapeutic effect of Cyn against GA by detecting inflammatory factors. We extracted and transcribed RNA from the treated BMDMs and fresh mouse hind paws and then conducted qRT-PCR to analyze gene expression. The results revealed higher mRNA expression of IL-1β, IL-6, iNOS, and TNF-α in the MSU and MSU+Cyn groups than in the PBS group and significantly lower expression in the MSU+Cyn group than in the MSU group (Figure 5(b–i)). These findings indicated that Cyn treatment reduced inflammatory factor production in mice with GA.

**Figure 5.** The effect of Cynarin on BMDMs and inflammatory factors. (a) CCK-8 kit detected the effect of Cyn on BMDMs. (b-e) After BMDMs were processed, the relative expression of inflammatory factors mRNA was detected. (f-i) After RNA extraction on the hind paws of mice, the relative expression of inflammatory factors mRNA was detected. Data were shown as mean ± standard deviation (SD) of three independent experiments. *p<0.05, **p<0.01, ***p<0.001 VS. MSU group or the group handled by LPS and MSU together. ^##^*p*<0.01, ^###^*p*<0.001 VS. PBS group or the group without LPS, MSU and Cyn.

### Cynarin inhibited the activation of NF-κB and JNK pathways and NLRP3 Inflammasome induced by MSU

We further clarified the action mechanism of Cyn in GA via western blot analysis of BMDMs and mouse hind paw tissues. Monosodium urate can activate the NF-κB and MAPK pathways and NLRP3 inflammasomes [22,27]. Therefore, we analyzed the effects of Cyn on the NF-κB, p38 MAPK, ERK1/2 MAPK, and JNK pathways and NLRP3 inflammasomes (Figure 6(a–g)). Cynarin inhibited the phosphorylation of IKKa/β, p65, and JNK in BMDMs induced with MSU, and the activation and production of NLRP3, Caspase 1, and IL-1β in hind paw tissues. We found that Cyn did not inhibit the phosphorylation of p38 and ERK1/2, but MSU activated them.

**Figure 6.** Cynarin inhibits the activation of NF-κB, JNK pathway and NLRP3 inflammasome induced by MSU. (a-j) Western blotting detected the protein levels of p-p38, p-ERK1/2, p-JNK, p-p65, p65, p-IKKa/β, Caspase1, NLRP3 and IL-1β, and analyzed these protein. Data were shown as mean ± standard deviation (SD) of three independent experiments. NS p>0.05, *p<0.05, **p<0.01, ***p<0.001 VS. the group handled by LPS and MSU together.

Western blotting revealed that that the average integrated density of p-p65, p-IKKa/β, p-JNK, NLRP3, Caspase 1, and IL-1β was significantly lower in the MSU+Cyn group than in the MSU group (Figure 6(b–d, h–j)). The average integrated density of p-p38 and p-ERK1/2 did not significantly change in the MSU+Cyn group when compared with that in the MSU group (Figure 6(e–f)). In brief, Cyn alleviated GA symptoms by inhibiting MSU to activate the NK-κB and JNK pathways and NLRP3 inflammasomes.

## Discussion

The compound Fu Rong Ye Babu ointment containing Centella Asiatica, Lithospermum, Folium Hibisci Mutabilis, Chixiaodou, and Cayratia japonica was initially screened via the Traditional Chinese Medicine Systems Pharmacology (TCMSP) database using the criteria of oral bioavailability > 30% and drug similarity > 0.18. Information on sitosterol, quercetin, and Cyn were extracted from the database. Quercetin has therapeutic effects against GA [29]. The effects of the remaining drugs were assessed using qRT-PCR, and finally Cyn was selected.

We found that Cyn had anti-swelling and anti-inflammatory effects in mice with GA. We used mouse models of GA to investigate the pharmacological effects of Cyn because the range of sources of Cyn is wide, its side effects are minimal, it is inexpensive, and Chinese herbal medicines or extracts are becoming more popular for treating GA [31–33]. Furthermore, Cyn is derived from the compound Fu Rong Ye Babu ointment, which is clinically effective in reducing GA swelling in patients.

We induced GA in mice using MSU because it causes deposition of urate crystals in the bones, joints, and other tissues where they cause damage and inflammation that finally progresses to GA [9,10]. Cynarin treatment reduced hind paw swelling in mice with GA within one week (Figure 2(a,b)). Ultrasound results further verified that Cyn treatment reduced swelling in these mice (Figures 2(c,d)). However, whether this anti-swelling effect was brought about through an anti-inflammatory process required further investigation. The drugs that are currently used to treat patients with GA can cause side effects, such as liver and kidney toxicity, and negatively impact treatment outcomes [23,34–36]. A morphological assessment of liver and kidney tissues from mice treated with Cyn revealed complete structures and obvious boundaries (Figure 3(a,b)). These findings indicated that Cyn does not adversely affect the liver and kidneys. However, whether Cyn affects other organs awaits further investigation.

Monosodium urate deposited in the tissues of patients with GA can cause a powerful inflammatory response [37,38]. Accordingly, we stained mouse hind paws with HE to analyze the effects of Cyn on inflammation. We found that Cyn inhibited infiltration by inflammatory cells (Figure 4a–c), including macrophages that play key roles in the onset of GA [39]. F4/80 and iNOS are markers of M1 macrophages [30,40]. Double immunofluorescence staining of the hind paws with anti-F4/80 and anti-iNOS primary antibodies revealed that Cyn inhibited M1 macrophage infiltration (Figure 4(d–e)).

We assessed the effects of Cyn on the viability of BMDMs stimulated with LPS and MSU *in vitro* [29]. The results of CCK-8 assays revealed that Cyn (290 μM) did not affect BMDMs viability (Figure 5(a)). Monosodium urate injection results in release of the inflammatory cytokines IL-1β, TNF-α, and IL-6 *in vivo*, and the M1 type macrophages produce iNOS and other inflammatory cytokines *in vitro* [28,41,42]. We assessed the expression of inflammatory factors using qRT-PCR. The results showed that Cyn inhibited production of the inflammatory factors IL-1β, IL-6, TNF-α, and iNOS (Figure 5(b–i)). The NF-κB and MAPK pathways and NLRP3 inflammasomes are activated by MSU [22]. We further confirmed the action mechanism of Cyn via western blotting. The results showed that Cyn inhibited activation of the NF-κB and JNK pathways as well as NLRP3 inflammasomes induced by MSU, but did not affect the p38 MAPK and ERK1/2 MAPK pathways (Figure 6(a-j)).

In summary, Cyn exerted anti-inflammatory and anti-swelling effects in model mice with GA induced by MSU crystals, through regulating the NF-κB and JNK pathways and NLRP3 inflammasomes. In other words, Cyn inhibited the MSU activation NF-κB and JNK pathways and NLRP3 inflammasomes and reduced the production of inflammatory factors, thereby alleviating inflammation and swelling. Small nucleolar RNA host gene 8 (SNHG8) accelerates the development of acute GA by upregulating adaptor related protein complex 3 subunit delta 1 (AP3D1) [8]. However, they did not consider the impact on specific types of cells and did not further analyze specific pathways. Our findings have enriched the understanding of GA research pathways and treatment strategies. However, the specific target(s) of Cyn remain to be elucidated.

## Conclusion

In summary, the study indicated that Cyn suppressed gouty arthritis induced by monosodium urate crystals by regulating NF-κB, JNK pathways and NLRP3 inflammasomes. Cynarin can be used as a clinical potential drug.
